# Comprehensive Analysis of Differentially Expressed circRNAs Reveals a Colorectal Cancer-Related ceRNA Network

**DOI:** 10.1155/2020/7159340

**Published:** 2020-09-01

**Authors:** Feng Que, Hua Wang, Yi Luo, Li Cui, Lanfu Wei, Zhaohong Xi, Qiu Lin, Yongsheng Ge, Wei Wang

**Affiliations:** ^1^Department of Colorectal Surgery, Affiliated Hospital of Integrated Traditional Chinese and Western Medicine, Nanjing University of Chinese Medicine, 210028 Nanjing, Jiangsu, China; ^2^Jiangsu Province Academy of Traditional Chinese Medicine, 210028 Nanjing, Jiangsu, China; ^3^Department of Oncology, Affiliated Hospital of Integrated Traditional Chinese and Western Medicine, Nanjing University of Chinese Medicine, 210028 Nanjing, Jiangsu, China; ^4^Key Laboratory of New Drug Delivery System of Chinese Materia Medica, Affiliated Hospital of Integrated Traditional Chinese and Western Medicine, Nanjing University of Chinese Medicine, 210028 Nanjing, Jiangsu, China; ^5^Department of Gastroenterology, Affiliated Hospital of Integrated Traditional Chinese and Western Medicine, Nanjing University of Chinese Medicine, 210028 Nanjing, Jiangsu, China

## Abstract

The morbidity and mortality of colorectal cancer (CRC) remained to be very high worldwide. Recently, circRNAs had been revealed to have a crucial role in cancer prognosis and progression. Numerous researches have shown that RNA sequencing technology and in silico method were widely used to identify pathogenic mechanisms and uncover promising targets for diagnosis and therapy. In this study, these methods were analyzed to obtain differentially expressed circRNAs (DECs). We identified upregulated 316 circRNAs and reduced 76 circRNAs in CRC samples, in comparison with those in normal tissues. In addition, a competitive endogenous network of circRNA-miRNA-mRNA was established to predict the mechanisms of circRNAs. Bioinformatics analysis revealed that these circRNAs participated in metabolism regulation and cell cycle progression. Of note, we observed the hub genes and miRNAs in this ceRNA network were associated with the survival time in CRC. We think this study could provide potential prognostic biomarkers and targets for CRC.

## 1. Introduction

The morbidity and mortality of colorectal cancer (CRC) remained to be very high worldwide [1, 2]. Over the past 10 years, great progress has been made in CRC prevention, diagnosis, and treatment [3]. Nevertheless, the prognosis of CRC is still poor [4]. It is therefore of importance to understand the mechanisms affecting CRC pathogenesis.

circRNAs are different from linear RNAs, which have a 5′ cap and 3′ tail structure [5]. circRNAs are characterized by forming a covalent closed-loop structure in the absence of 5′-3′ polarity or polyadenylated tails [6]. More and more researches have shown that circRNAs are a sort of affluent, miscellaneous, and conservative RNA molecules [7, 8]. Of note, up-and-coming evidences suggested that circRNAs modulated various biological processes, such as cell viability, differentiation, apoptosis, and angiogenesis [9, 10]. Presently, numerous researches have revealed that circRNAs are dysregulated in various carcinomas, implying that circRNAs displayed an important role in the occurrence and development of human carcinomas. With the development of high throughput RNA sequencing and bioinformatics methods, the advantage of circRNAs emerged gradually. Currently, some researches had shown that circRNAs modulated alternative splicing and gene expression level through sponging microRNAs (miRNAs) [11, 12]. At the same time, disorders of circRNAs took part in carcinogenesis and cancer development of CRC [13, 14], liver cancer [15], and gastric cancer [16–19]. These findings indicated that circRNAs, as a new kind of endogenous noncoding RNA, have been a new hotspot in the cancer research and probably would exhibit important functions in the development of tumor.

mirRNAs are a member of noncoding RNAs with approximate 22 nucleotides in length [20, 21]. mirRNAs exhibit inhibitory function on target gene expression via miRNA response elements (MREs) in the 3-UTR of transcripts [22]. Several researches had revealed that circRNAs sponged miRNAs by binding to corresponding MREs in many diseases, which has also been identified in the occurrence and development of cancer as previously described [23, 24]. Numerous evidences showed that circRNAs, exhibiting as miRNAs spongers, could modulate CRC growth, progress, and metastasis [25, 26]. For example, ciRS-7 sponged miR-7 and suppressed target gene expression in many tumors, including CRC [26]. Additionally, circHIPK3 probably displayed as miR-1207/miR-637/miR-7 sponge and retarded its antitumor function, thereby promoting CRC cell viability [27–29]. hsa_circ_0091074 modulated TAZ level by microRNA-1297 in breast cancer cell [30]. CircSMC3 modulated tumor genesis of gastric cancer via targeting miR-4720-3p/TJP1 axis [31]. In colon cancer, hsa_circ_0055625 deriving from the expression profile of circRNAs promoted colon cancer cell viability via sponging miR-106b-5p [32]. hsa_circ_0007843 was a sponger of miR-518c-5p and modulated colon cancer cells migration and invasion [33]. Nevertheless, further researches are still needed to investigate the probable mechanisms of tumorigenesis, might aid in the diagnosis and treatment of CRC, and may be of help for CRC diagnosis and treatment.

In our study, we systematically assessed circRNA expression in 3 paired CRC and normal tissues. We discovered that the expression profile of circRNAs was dramatically distinct between CRC and normal tissues. Meanwhile, we constructed a circRNA-miRNA regulatory network in CRC. Our data suggested that circRNAs were linked to CRC occurrence and development, thus supplying more long-range perspective indicators and new biomarkers for CRC.

## 2. Materials and Methods

### 2.1. Samples

This study got approval from The Ethics Review Board of Affiliated Hospital of Integrated Traditional Chinese and Western Medicine, Nanjing University of Chinese Medicine. All CRC patients signed written informed consent. A total of 3 paired CRC and normal were used in this study.

### 2.2. Construction and Sequencing of RNA Library

Whole RNA was harvested by TRIzol reagent (Invitrogen, CA, USA) as manually described and then subjected to detect quality and concentration of purified RNA by Bioanalyzer 2100 (Agilent, CA, USA) and Qubit 2.0, respectively.

The library of circRNA was established referring to the instruction of the NEBNext Ultra Small RNA Sample Library Preparation Kit of Illumina. RNase R was applied to digest linear RNA, and rRNA probe was used to remove rRNA accordingly. The first strand is synthesized using stochastic hexapolymers and templates of circRNA. Subsequently, the second strand of cDNA was completed. AMPure XP beads were applied to make purification of lncRNAs and circRNAs. T4 DNA polymerase and Klenow DNA polymerase could attain the goal of the blunt end of DNA. Poly(A) tail was added into 3′ end of DNA and then sequenced. AMPure XP beads were applied to choose the size of fragments. USER enzyme was used to degrade the second strand comprising cDNA. The library of ncRNAl and circRNA was obtained by PCR amplification. Finally, the libraries were subjected to paired-end sequencing with pair end 150 bp reading length on an Illumina HiSeq sequencer (Illumina, San Diego, CA, USA) according to a previous report [34].

Differentially expressed circRNAs (DEC) between cancer and normal tissue were identified with defined threshold values > 1.0 (∣logFC | >1) and *p* values < 0.01 (*p* value < 0.01).

### 2.3. Construction of Competing Endogenous (ceRNA) Network

The CSCD database (http://gb.whu.edu.cn/CSCD) was applied to predict MREs, RNA-binding proteins (RBPs), and open reading frames (ORFs) [35]. The links between miRNAs and the circRNAs or mRNAs were forecasted by a ceRNA network. The interplay between mRNA and miRNA, of which sequences and interpretation were derived from miRBase [36], was forecasted by miRTarbase [37], TargetScan [38], and miRDB [39]. The ceRNA network comprising target genes of miRNA and circRNAs was established utilizing Cytoscape software (version 3.6.1) [40].

### 2.4. Bioinformatics Analysis

GO (http://www.geneontology.org) was applied to identify and annotate the sequences of homologous genes and proteins in a variety of organisms, which can help us clarify the particular role of specified genes.

The KEGG (http://www.genome.jp/kegg/) [41] database was used to predict the potential pathways regulated by candidate mRNAs or circRNAs. Adjusted *p* < 0.05 and *q* < 0.05 represented obvious annotations of enriched function of circRNAs.

### 2.5. Statistical Analysis

GraphPad Prism software version 6 (GraphPad Software, Inc.) was applied for data processing. The represented data obtained from at least three independent experiments in triplicates was shown as the mean ± SD. Two-tailed paired Student's *t*-test was applied to compare two groups. The overall survival curve was generated using the Kaplan–Meier method and the log-rank test. Significant difference was shown as *p* < 0.05.

## 3. Results

### 3.1. Identification of DECs in CRC

RNA sequencing was applied to determine the expression profile of circRNAs in 3 CRC and normal tissues. Hierarchical clustering, as one of most extensive clustering analysis toolsets, was applied to assess gene expression data (Figure 1(a)). The difference between normal and CRC samples was visualized by the volcano plot. The vertical lines indicated approximate 2.0-fold, and the horizontal lines suggested a *p* value of 0.05. Red dots included in the indicated figures represented the differentially expressed circRNA, meaning significant difference (Figure 1(b)). In our results, compared with normal tissues, 316 circRNA expression level was increased and 76 circRNA expression level was reduced.

Of note, some of these circRNAs had been demonstrated to be related to cancer progression. For example, hsa_circ_0084663 was validated to be related to sorafenib-resistant liver cancer [42]. Very interestingly, we found that hsa_circ_0061776 and hsa_circ_0006528 were also upregulated in colon samples by analyzing the supplementary table in an independent report [25]. Meanwhile, we found these different expressed circRNAs could be divided into 8 clusters. As shown in Figure 1, subcluster 1 included 188 circRNAs (Figure 1(c)), subcluster 2 included 33 circRNAs (Figure 1(d)), subcluster 3 included 19 circRNAs (Figure 1(e)), subcluster 4 included 43 circRNAs (Figure 1(f)), subcluster 5 included 21 circRNAs (Figure 1(g)), subcluster 6 included 33 circRNAs (Figure 1(h)), subcluster 7 included 42 circRNAs (Figure 1(i)), and subcluster 8 included 13 circRNAs (Figure 1(j)).

### 3.2. The Function Prediction of the Host Genes of circRNAs

Previous studies had showed that circRNAs may play its roles in human diseases via their host genes. Thus, the potential functions of the host genes were assessed by GO and KEGG. The host genes of DECs are enriched in GO terms including primarily contained organization of cellular component or biogenesis, cell cycle, miRNAs (mainly for gene silencing), mitotic cell cycle, cell cycle process, and posttranscriptional gene silencing by RNA. The host genes of DECs are enriched in CC terms, including cytosol, organelle, cytoplasm, membrane-less organelles, intracellular membrane-less organelles, and nucleus. The differentially expressed genes are enriched in molecular function term and protein binding (Figure 2(a)).

Through KEGG analysis, the function of the host genes of DECs participated in modulating signaling pathways, including adherent junction, VEGF signaling pathway, thyroid cancer, endometrial cancer, serotonergic synapse, leukocyte transendothelial migration, bacterial invasion of epithelial cells, non-small cell lung cancer, and long-term depression (Figure 2(b)).

### 3.3. Construction of a circRNA-miRNA-mRNA Network

Numerous evidences showed DECs could competitively sponge miRNAs and then suppressed downstream genes of miRNAs. In the present study, we used an integrated database, CSCD, to predict the interaction between miRNAs and circRNAs. Then, the specific mRNA-miRNA interactions were identified using miRTarBase, TargetScan, and miRDB. The network was constructed by Cytoscape. As presented in Figure 3, a total of 41 miRNAs, 166 circRNAs, and 2427 mRNAs were included in this ceRNA network (Supplementary table 1).

From the network, 6 circRNAs (hsa_circ_0004841, hsa_circ_0007523, hsa_circ_0008038, hsa_circ_0000799, hsa_circ_0002744, and hsa_circ_0005620) were found to be linked to more than 10 different miRNAs, which were identified as key circRNAs in CRC. Meanwhile, 14 mRNAs (including QKI, HECTD2, SYNCRIP, RUNX1, SEMA6D, VCL, MBNL1, HMGA2, ABCC5, ARRDC4, CPD, JPH1, MTDH, and TP53INP1) were identified as key regulators in this network, which were targeted by more than 25 miRNAs. In addition, hsa-miR-93-5p, hsa-miR-20a-5p, hsa-miR-17-5p, hsa-miR-106a-5p, hsa-let-7b-5p, hsa-miR-27a-3p, hsa-miR-15a-5p, hsa-miR-16-5p, hsa-let-7c-5p, hsa-miR-103a-3p, hsa-let-7d-5p, hsa-miR-107, hsa-let-7e-5p, hsa-miR-23a-3p, hsa-let-7a-5p, hsa-miR-30a-5p, hsa-miR-19a-3p, and hsa-miR-19b-3p were identified as the key miRNAs by targeting more than 500 genes.

### 3.4. GO and KEGG Pathway of ceRNA Network

Considering the above DECs, the functional role was still unclear, and the function of circRNA was predicted with their targeting mRNAs. GO and KEGG pathway analyses of differentially expressed mRNAs with significance were conducive to understand circRNAs.

The data showed that the target gene function of circRNAs was related to the modulation of metabolism, energy pathways, cell growth and/or maintenance, transport, cell communication, signal transduction, nucleobase regulation, nucleoside, nucleotide and nucleic acid metabolism, cell cycle, apoptosis, gene expression regulation, epigenetics, cell motility, enzyme activity negative regulation, DNA replication, lipid metabolism, chromosome segregation, and steroid metabolism (Figure 4(a)).

KEGG pathway analysis results revealed the target genes of circRNAs were related to the pathways, including syndecan-1-mediated signaling events, glypican pathway, nectin adhesion pathway, TRAIL signaling pathway, glypican 1 network, integrin family, ErbB receptor signaling network, VEGF and VEGFR signaling network, proteoglycan syndecan-mediated signaling events, LKB1 signaling events, mesenchymal-to-epithelial transition, and epithelial-to-mesenchymal transition (Figure 4(b)).

### 3.5. The Dysregulation of Hub Genes and miRNAs Was Correlated to the Survival Time in Patients with CRC

Then, to further explore the functions of these hub genes in the network in carcinogenesis and the development of CRC, we analyzed the correlation between the expression of hub mRNAs, or miRNAs and survival time in patients with CRC using GEPIA [43] and Kaplan–Meier plotter database. Unfortunately, both databases do not contain circRNAs. Thus, we did not analyze the correlation between the survival time and the expression of circRNAs in CRC. As shown in Figure 5, the Kaplan–Meier curves indicated that higher expressions of QKI (Figure 5(a)), ABCC5 (Figure 5(b)), RUNX1 (Figure 5(c)), CALD1 (Figure 5(d)), and CLIP4 (Figure 5(e)) were dramatically linked to poorer overall survival. However, overexpressions of SYNCRIP (Figure 5(f)) and SEMA6D (Figure 5(g)) were related to longer survival time in patients with CRC.

Meanwhile, as presented in Figure 6, the Kaplan–Meier curves showed that hsa-miR-20a (Figure 6(a)), hsa-let-7b (Figure 6(b)), and has-miR-15 (Figure 6(c)) were related to longer survival time in patients with CRC. However, the higher expression level of hsa-let-7d (Figure 6(d)) would result in shorter overall survival time. All the results demonstrated that dysregulation of hub genes and miRNAs could be the potential targets for the prognosis of CRC.

## 4. Discussion

RNA sequencing technology has made it possible to extensively explore gene expression and promoted the study of susceptibility to disease, which is beneficial for disease treatment at the molecular level. Numerous researches have shown that RNA sequencing technology and in silico method were widely used to identify pathogenic mechanisms and uncover promising targets for diagnosis and therapy [44–46].

In this study, the RNA sequencing was applied and the bioinformatics data was analyzed to obtain differentially expressed circRNAs (DECs). Then, the probable DEC-sponged miRNAs was identified by Cancer-Specific CircRNA Database (CSCD). In addition, target mRNAs were predicted by bioinformatics analysis and a competitive endogenous network of circRNA-miRNA-mRNA was established. Gene ontology (GO) and Kyoto Encyclopedia of Genes and Genomes (KEGG) databases were applied to analyze candidate mRNAs and then assume the signaling pathways underlying in CRC. To identify DECs and explore the hidden mechanisms in this study might be helpful to develop novel treatment for CRC.

Here, we systematically analyzed and compared the expression profile of circRNAs in 3 CRC and normal tissues. The data suggested that circRNA expression profile was largely distinct in CRC tissues, compared to that in normal tissues. Notably, 289 of circRNAs expression presented ectopic in CRC after comparison with those in normal tissues. 76 of circRNA expression level were reduced, and 316 of circRNAs expression level were induced in CRC. We also observed this interesting phenomenon. We found the number of upregulated circRNAs is more than 3-fold compared to the number of downregulated circRNAs. Very interestingly, multiple previous studies also reported this phenomenon. For example, He et al. identified 94 downregulated circRNAs and 28 upregulated circRNAs in gastric cancer with GSE89143 [47] and identified 144 downregulated circRNAs and 52 upregulated circRNAs with GSE78092 [48]. Shi et al. observed 469 upregulated circRNAs and 275 downregulated circRNAs in ESCC [49]. Wen et al. found 109 circRNAs that were significantly upregulated and 56 circRNAs that were downregulated among the rheumatoid arthritis patients by using RNA-seq method [50]. Our findings together with previous reports showed the circRNA expression pattern between disease and nondisease samples was not similar with mRNAs and lncRNAs, suggesting that posttranscriptional regulation may have a crucial role in modulating circRNA formation. The function of circRNAs in the host participated in modulating cell cycle, gene silencing by miRNA, mitotic cell cycle, cell cycle process, and posttranscriptional gene silencing by RNA.

Recently, the links between noncoding RNAs and cancer were greatly investigated. Newly generated researches showed that noncoding RNAs displayed importance in carcinogenesis and cancer development [51]. Some reports have shown that circRNAs displayed importance in the process of biology and the progression of diseases through sponging miRNA [13, 14]. For example, circular RNA Circ100084, exhibiting as the sponge of miR-23a-5p, modulated the expression of IGF2 in hepatocarcinoma [52]. In this study, a total of 41 miRNAs, 166 circRNAs, and 2427 mRNAs were included in this ceRNA network. Bioinformatics analysis showed that the function of circRNA target genes had an association with metabolism regulation, energy pathway regulation, cell growth and/or maintenance, transport, cell communication, signal transduction, nucleobase regulation, nucleoside, nucleotide and nucleic acid metabolism, cell cycle, apoptosis, gene expression regulation, epigenetics, cell motility, enzyme activity negative regulation, DNA replication, lipid metabolism, and chromosome segregation.

In the present study, 14 mRNAs (including QKI, HECTD2, SYNCRIP, RUNX1, SEMA6D, VCL, MBNL1, HMGA2, ABCC5, ARRDC4, CPD, JPH1, MTDH, and TP53INP1) were identified as primary regulators in this network, which were targeted by more than 25 miRNAs. Several reports had illustrated the key characters of these mRNAs in human cancers as previously described. QKI protein has been revealed in human and was associated with many human diseases, such as cancer, and neurological diseases, such as human hereditary ataxia, various sclerosis, or schizophrenia. Currently, several findings suggested that knockout of QKI-5 genome would result in increased cell viability and dedifferentiation in cancers, indicating that QKI-5 was an inhibitor of tumor in multiple types of many cancers [53]. QKI was identified as a key regulator of alternative splicing in cancers. Very interestingly, QKI was found to be related to the formation of circRNAs. Ablated QKI led to arrestment of circRNA expression-related EMT [54]. Further reports confirmed the active roles of QKI during the biogenesis of circRNAs [54]. Studies towards solid tumors have indicated RUNX1 possessing a context-dependent function displayed as an oncogene or a suppressor of tumor. These functions of Runx1 have been shown in breast, prostate, lung, and skin cancers, presenting a relationship between different subtypes of cancers and stages of tumor progress. There are more and more evidences showing that Runx1 inhibited the invasiveness of most kinds of breast cancer, especially in the early stage of tumor development. In colon cancer, Systems Pharmacogenomics identified RUNX1 as an aspirin-responsive transcription factor. Vinculin (Vcl), a 117 kDa membrane-related protein, was expressed in global cells and functioned importantly in mechanotransduction. MBNL1, a RNA-binding protein, bind to 3′UTRs and facilitate mRNA decay. Hence, HMGA2 is considered to be an oncogene, which serves as a critical regulator of proliferation and survival. Besides, HMGA2 overexpression is linked to initial of metastasis and poorly prognostic status in a large number of cancers types [55]. ABCC5, also named by multidrug-resistance protein 5, has been shown to transport nucleosides and antifolates. The enhanced ABCC5 level was shown to be related to the occurrence of breast cancer, hepatocellular carcinoma, and pancreatic ductal adenocarcinoma. What is more, MTDH has been demonstrated to function vitally in tumor genesis, development, and resistance to chemotherapy. The abnormal expression and dysfunction of MTDH are related to the viability, survival, and metastasis of tumor cells. Apoptotic protein TP53INP1 (tumor protein 53-inducible nuclear protein 1) participated in the response from cellular stress.

Here, we identified 18 key miRNAs involved in regulating the activity of circRNAs. Among these miRNAs, higher expression of hsa-miR-20a, has-Let-7b, and hsa-miR-15 but lower expression of has-Let-7d were related to longer survival time in CRC. The miR-20a expression level was raised in CRC patients after a comparison with that in control. Several recent studies demonstrated that miR-20a retarded autophagy induced by hypoxia through targeting ATG5/FIP200 in CRC and modulated the sensitivity of CRC cells to NK cells by targeting MICA. Universal ablation of miR-15 (microRNA 15) and miR-16 in cell lines and tissues of numerous cancers revealed that the function of miR-15a/16-1 exhibited vitally in the progression of tumor. The prospect of miR-15a/16-1 was herein noteworthy in cancer therapy. In colon cancer, upregulation of miR-15a hindered cell viability and cycle. In normal cells, let-7 modulated cell viability, cycle, apoptosis, metabolism, and stemness. However, the let-7 microRNA level in CRC was shown to be decreased and was taken as a suppressor of tumor.

There are some limitations in our research. Firstly, the amount of samples is not sufficient. Secondly, our results merely from present toolsets and databases needed to be further improved. Thirdly, the parameter of prognosis regarding DEcircRNAs in CRC should be identified. More clinical samples and experiments would be supplemented in the following studies to consolidate our conclusions and evaluate the characters of these DEcircRNAs.

In conclusion, the present study identified 316 upregulated circRNAs and 76 downregulated circRNAs in CRC samples, in comparison with those in normal tissues. Bioinformatics analysis revealed that these circRNAs participated in metabolism regulation and cell cycle progression. Furthermore, we constructed differently expressed circRNAs to regulate ceRNA networks based on RNA-seq methods and bioinformatics analysis. Finally, we thought our study could provide novel biomarkers and insights for CRC prognosis.

## Figures and Tables

**Figure 1:** Identification of DECs in CRC. (a) Hierarchical clustering identified differently expressed circRNAs in CRC. (b) The volcano plot showed differently expressed circRNAs in CRC. (c) Subcluster 1 included 188 circRNAs. (d) Subcluster 2 included 33 circRNAs. (e) Subcluster 3 included 19 circRNAs. (f) Subcluster 4 included 43 circRNAs. (g) Subcluster 5 included 21 circRNA. (h) Subcluster 6 included 33 circRNAs. (i) Subcluster 7 included 42 circRNAs. (j) Subcluster 8 included 13 circRNAs.

**Figure 2:** The function prediction of the host genes of circRNAs. (a) The GO analysis of the potential functions of the host genes of DECs. (b) The KEGG pathway analysis of the potential functions of the host genes of DECs.

**Figure 3:** Construction of a circRNA-miRNA-mRNA network. A total of 41 miRNAs, 166 circRNAs, and 2427 mRNAs were included in this ceRNA network.

**Figure 4:** GO and KEGG pathway analysis of ceRNA networks. (a) The GO analysis of the potential functions of ceRNA networks. (b) The KEGG pathway analysis of the potential functions of ceRNA networks.

**Figure 5:** The dysregulation of hub genes was correlated to the survival time in patients with CRC. The Kaplan–Meier curves indicated that higher expression of QKI (a), ABCC5 (b), RUNX1 (c), CALD1 (d), and CLIP4 (e) and lower expression of SYNCRIP (f) and SEMA6D (g) were dramatically linked to poorer overall survival in patients with CRC.

**Figure 6:** The dysregulation of hub miRNAs was correlated to the survival time in patients with CRC. The Kaplan–Meier curves indicated that higher expression of hsa-miR-20a (a), hsa-let-7b (b), and has-miR-15 (c) and lower expression of hsa-let-7d (d) were dramatically linked to longer overall survival in patients with CRC.

## Data Availability

The datasets used during the present study are available from the corresponding author upon reasonable request.

## Supplementary Materials

Supplementary Materials Supplementary table 1: the detailed information about circRNA-miRNA-mRNA network.
